# Mathematical Modeling and Nail Placement Accuracy Analysis of NF-1 Neurofibromatosis Scoliosis

**DOI:** 10.1155/2022/4229377

**Published:** 2022-01-31

**Authors:** Guangxuan Yan, Jincai Yang, Shibing Qin, Peng Yin, Aixing Pan, Yong Hai

**Affiliations:** ^1^Department of Orthopedics, Beijing Chest Hospital, Capital Medical University, Tongzhou District, Beijing 101149, China; ^2^Department of Orthopedics, Beijing Chaoyang Hospital, Capital Medical University, Chaoyang District, Beijing 100020, China

## Abstract

We have analyzed the arch root morphology, nail placement accuracy, degree of arch deformity, and three-dimensional Cobb angle in patients with NF scoliosis by CT 3D reconstruction. Likewise, we have thoroughly examined arch root morphology, nail placement accuracy, degree of arch deformity, and three-dimensional Cobb angle in patients with idiopathic scoliosis by CT 3D reconstruction. The results of the two groups were statistically analyzed and compared to assess the efficacy and other morphological differences between these groups. For this purpose, 276 patients with scoliosis, including 221 with idiopathic scoliosis and 16 with neurofibromatosis scoliosis, were treated in the hospital, which is from May 2008 to December 2016. The 16 patients with idiopathic scoliosis were matched with patients with neurofibromatosis, and the postoperative CT data were reconstructed in three dimensions, and the measurements included arch morphology, arch transverse diameter, arch-rib joint transverse diameter, three-dimensional coronal Cobb angle, and correction rate. The data of the two groups were statistically analyzed to compare the arch morphology, nail placement accuracy, and treatment effect between patients with NF and patients with AIS. Statistical analysis was performed to compare the differences between NF and AIS patients in terms of morphology, nail placement accuracy, and treatment outcome. The results showed that there were more severely deformed pedicles in NF patients than in idiopathic scoliosis, and the difference between them was statistically significant. Of the 142 screws placed in the NF group, 88 screws were in a good position, and the remaining 54 screws were misplaced.

## 1. Introduction

Neurofibromatosis is a relatively rare and complex autosomal dominant disease, mostly thought to be associated with mutations in the neurofibromatosis suppressor gene [1], and often manifests cellularly as an abnormal proliferation of neural crest cells, which are important constituent cells during the establishment of the neural tube, and they are able to migrate to various parts of the embryo and differentiate into the appropriate tissues and cells. Externally, almost all patients with neurofibromas have skin pigmentation (including milk coffee spots, skin freckles, and Lisch nodules) and neurofibromas in the skin and subcutis. Some patients also develop skeletal abnormalities (scoliosis deformities, tibial pseudarthrosis), brain tumors (benign meningiomas or even malignant gliomas), peripheral nervous system tumors (intralesional neurofibromas, plexiform fibromas, malignant peripheral nerve sheath tumors), cognitive impairment, and behavioral disturbances that lead to poor social integration and even serious physical health problems [2, 3]. The current literature tends to classify neurofibromas into 2 types: Neurofibromatosis type I (NF1) and Neurofibromatosis type II (NF2). Type II is less common and is mainly characterized by bilateral auditory neuromas with minimal skeletal effects; therefore, in this paper, patients with neurofibromatosis I usually have abnormal bone metabolism, abnormal spinal development such as flattened vertebrae, wedge-shaped vertebral body, narrowed pedicles, enlarged intervertebral foramina, and rib protrusion into the spinal canal, resulting in scoliosis deformity [4], with an incidence of 10%–60%. 10%–60% is the most common skeletal change in patients with NF [5]. Of all the causes of scoliosis, neurofibroma as a cause, Rezaian et al. concluded that only about 3%. Idiopathic scoliosis is the most common cause of scoliosis; these patients have essentially no abnormal bone development and the pathological curvature is often caused by neuromuscular dysfunction, which accounts for about 80% of the total causes of scoliosis. Congenital scoliosis means that the bony structures are abnormal at birth, such as hemivertebrae deformity, butterfly vertebrae, cuneiform vertebral changes, or poor spinal segmentation: fused vertebrae lead to scoliosis deformity. In addition, there are some special types of scoliosis, such as neuromuscular scoliosis, Marfan syndrome, and other interstitial diseases caused by scoliosis, osteochondral dyskinesia combined with scoliosis, and rickets; after spinal trauma, inflammatory tumors of the paravertebral canal can cause scoliosis.

In addition to deformity affecting appearance and movement, symptoms such as pain, lower extremity numbness, lower extremity weakness, and urinary disturbance cauda equina compression are also the reasons why patients are seen, often because of a deformed spine or a paravertebral neurofibroma compressing the spinal canal and nerve roots inward [6]. The best imaging method to detect neurofibromin scoliosis is CT. Pencil-like changes of the ribs and protrusion of the ribs into the spinal canal are rare but dangerous signs that can only be detected by CT, and preoperative CT can detect arch deformities of the spine, absence of the arch, and bulging of the spinal membrane. It is also possible to reconstruct the vertebral body after surgery to evaluate the surgical results and summarize the experience. Therefore, in this paper, we hope that 3-dimensional reconstruction can provide a more visual and accurate measurement of the efficacy indexes. It has been reported in the literature that MRI can more accurately detect paravertebral soft tissue masses and exclude the possibility of malignant peripheral nerve sheath tumors [7, 8], which are difficult to distinguish with CT. Because of the lack of awareness of neurofibromas and malignant peripheral nerve sheath tumors, some experts believe that PET should be performed if there are indistinguishable paravertebral masses [9]. Protrusion of ribs into the spinal canal is a rare but serious imaging manifestation, which has been reported in many papers [10–12], and others, such as vertebral arch deformities, reduced vertebral bone mass, and bulging spinal membranes in the spine, have significant implications for pedicle nailing and internal fixation. When inserting pedicle screws, if the 3-dimensional position of the spine is neglected, poor development of the pedicle often leads to dangerous nail placement or even dural tear, which is a common factor for postoperative neurological deficits; unlike patients with idiopathic scoliosis, patients with NF have severe deformity and are more likely to have dangerous nail placement. In this paper, we will try to compare the screw misplacement rate of NF-related scoliosis with that of idiopathic scoliosis patients.

Treatment options for neurofibromatosis scoliosis are similar to idiopathic scoliosis, so it is also called idiopathic-like, but also different. Treatment of neurofibromatosis scoliosis is similar to idiopathic scoliosis, without the combination of other systemic diseases. Patients with scoliosis less than 20° are recommended for observation and treatment. Patients with scoliosis of more than 40° usually undergo posterior orthopedic internal fixation, and for patients with scoliosis of more than 55°, simultaneous anterior release graft fusion and posterior internal fixation are preferable due to the greater stiffness of the spine in patients with NF [13].

With the continuous progress of computer computing speed and calculation methods in the past decade, the previous method of counting the arch root morphology and nail placement accuracy by CT tomography and PACS of MR faces the disadvantages of not being accurate and not being three-dimensional and intuitive enough. In this paper, we use Materialise'S Interactive Medical ImageControlSystem (Mimics) software, which is widely used in clinical practice. Mimics can obtain a 3D reconstruction model of the target, analyze the data through measurement software, and guide the postoperative summary. Mimics can obtain a 3D reconstruction model of the target, analyze the data through measurement software, and guide the postoperative summary, which is more accurate than the data collection and processing of traditional CT and PACS medical imaging systems. In this paper, we will use Mimics software to obtain satisfactory 3D reconstructed images to reflect changes in spinal deformity indicators, the accuracy of nail placement, and other indicators that are difficult to accurately reflect with traditional PACS systems. The DICOM files obtained from Siemens Somatom Sensation 64-layer spiral CT scan samples were processed by Mimics17.0l software and imported into 3-matic 9.0 software to generate 3D models for multiple data measurements and nail placement accuracy analysis from any angle and any plane and computed on the computer to increase the accuracy of measurements Reducing errors [14].

In this paper, we have analyzed the arch root morphology, nail placement accuracy, degree of arch deformity, and three-dimensional Cobb angle in patients with NF scoliosis by CT 3D reconstruction. Likewise, we have thoroughly examined arch root morphology, nail placement accuracy, degree of arch deformity, and three-dimensional Cobb angle in patients with idiopathic scoliosis by CT 3D reconstruction. The results of the two groups were statistically analyzed and compared to assess the efficacy and other morphological differences between these groups. For this purpose, 276 patients with scoliosis, including 221 with idiopathic scoliosis and 16 with neurofibromatosis scoliosis, were treated in the hospital, which is from May 2008 to December 2016.

The remaining portions of this article are organized as follows.

In the subsequent section, a brief, but thorough, review of the existing literature is presented where the focus is on sepsis-related diseases. In Section 3, the proposed mechanism is presented where sophisticated detail is provided about various parts of the proposed setup. Experimental results and observations were presented in Section 4 of this manuscript. Finally, concluding remarks and future directives are provided in the last section.

## 2. Materials and Methods

### 2.1. Research Equipment

64-row spiral dual-source CT GE, USA, was provided by the Department of Radiology, The First Affiliated Hospital of Guangxi Medical University.

### 2.2. Research Software

AW Volumeshare 2 Computer Operating System Materialise'S Interactive Medical System3-matic was provided by General France Materialise, Belgium.

### 2.3. Research Subjects

A total of 276 patients with scoliosis treated in our hospital from May 2008 to December 2016 were collected by checking the medical record system, including 39 patients with congenital scoliosis, 221 patients with idiopathic scoliosis, and 16 patients with neurofibromatosis scoliosis. Among the 221 patients with idiopathic scoliosis, patients with similar age, sex, curvature, and surgical approach to the 16 patients with neurofibromatosis scoliosis were selected. Of these 32 patients, 14 were male and 18 were female; the mean age was 14.3 years (7 to 24 years). There were 16 cases of neurofibromatosis scoliosis with a mean scoliosis angle of 68.6.6° (46°–126°) and 381 of thoracolumbar pedicles, and 142 pedicle screws were inserted. In 16 cases with idiopathic scoliosis, 344 pedicles were inserted and 111 pedicle screws were inserted, and the surgical approach was posterior scoliosis orthopedic fusion and internal fixation, with preoperative X-ray, CT, and MRI examinations performed as usual. Postoperatively, they wore appropriate braces and were followed up regularly with dual-source CT and radiographs at the outpatient clinic.

### 2.4. Proposed Method of Diagnosis

Criteria for neurofibromatosis scoliosis according to those developed at the 1987 National Institutes of Health (NIH) meeting [15] were as follows: (1) 6 or more milk coffee spots larger than 5 mm in diameter before puberty or milk coffee spots larger than 15 mm in diameter in adults; (2) two or more types of cutaneous subcutaneous neurofibromas or trabecular neurofibromas; (3) two or more types of subcutaneous neurofibromas or trapezoid neurofibromas; (3) pigmented freckles in the axilla or groin; (4) optic glioma; (5) 2 or more Lisch nodules (iris malformations); (6) significant skeletal changes such as pterygoid dysplasia and tibial pseudarthrosis; (7) NF in the immediate family. 2 or more of the above 7 items are diagnostic.

Idiopathic scoliosis criteria were as follows: absence of bony structural abnormalities, exclusion of congenital scoliosis, and other specific types of scoliosis. All 32 patients had a complete medical history, complete imaging data (X-ray, CT), and no other complications such as paravertebral tumors on imaging and were hospitalized in our spinal orthopedic surgery department between May 2008 and December 2016 and treated with posterior surgery.

A CT scanner was used for this study: the machine was provided by the radiology department of our hospital (Siemens Somatom Sensation 64CT). The scan layer thickness was 0.6 mm, and preoperative and postoperative cross-sectional images of the spine were obtained and saved in DICOM format on a personal computer for 3D digital reconstruction using Mimics 17.1 software. The reconstruction results were output in mcs format, which are shown in Figures 1 and 2.

1. Open Mimics 17.1 software, select Menu-File-New Project to import preoperative and postoperative CT images in DCM format, determine the anterior-posterior orientation, and click convert to generate.
2. Create a mask (New Mask command), click Thresholding to adjust the threshold value of the mask, the specific threshold value according to the parameters to be measured, including the threshold value of the nail bar system, and the threshold value of the bone part, try to remove metal artifacts, click Apply to determine.
3. The Crop Mask command and the erase function in Edit masks are used to separate the vertebral body from the ribs, sternum, etc., using clinical anatomy knowledge to preserve only the vertebral body, the pedicle, and other structures to be measured.
4. Select the established mask and click Calculate 3D from Mask to achieve the initial 3D reconstruction of the scoliosis spine simulation model.
5. Import the resulting image into 3D operation software, carry out Move, Rotate, and Rescale commands to adjust the 3D spatial position, and get a more detailed model.
6. Click on the smoothing option in the Tools above to smooth the result and improve the roughness and excessive noise in the image.
7. The above method was repeated for 32 patients with scoliosis, and measurements of pedicle fractionation, Cobb angle, and nail placement accuracy were performed on 3-dimensional images.

### 2.5. Observed Indicators

Arch root typing: Verma et al. have refined and added to Lenke's arch root typing [16]. The specific typing is as follows: type A (normal) with an internal diameter of ≥3 mm and a large cancellous canal, type B (narrow) with an internal diameter of <3 mm and a small cancellous canal, type C (isthmic sclerosis) with a cortical canal and an “*x*” shape of the internal and external walls, type D (complete sclerosis) with no cortical canal and a striated sclerotic arch, and the outer wall of the arch. Type D (complete sclerosis) has no cortical canal cavity, and the roots are sclerotic in the form of cords; the outer wall of the vertebral arch with the outer edge of the vertebrae has an I-shaped morphology; Type E has an absence of the vertebral arch [17].

Classification of screw misplacement: according to the evaluation method of Li et al. [18], screw penetration is divided into 4 levels by postoperative CT, and level 0: no penetration; Grade 1: penetration less than 25% of the screw diameter; Grade 2: penetration up to 25%–50% of the screw diameter; Grade 3: the penetration part greater than 50% of the screw diameter. Grade 0 and grade 1 are considered as correct screw placement, grades 2–4 are considered as screw misplacement, and the screw misplacement rate = the number of screws in grade 2–4/the total number of screws inserted × 100%; the satisfaction rate of screw placement =  number of grade 0-1 screw/total number of screws inserted × 100%. Correction rate of the main coronal curve: correction rate of the main coronal curve after the operation. Correction rate of main coronal curve = (Cobb angle of main coronal curve before operation − Cobb angle of main thoracic curve immediately after operation)/Cobb angle of the main coronal curve before operation) × 100％. Follow-up correction rate: the correction rate of the coronal plane of the main curve during the follow-up of 4–48 months. The follow-up correction rate = (Cobb angle of the coronal plane of the main curve before operation, Cobb angle of the coronal plane of the main thoracic curve during the last follow-up)/Cobb angle of the coronal plane of the main curve before operation) × 100%. Correction loss = coronal Cobb angle of main thoracic curvature at the last follow-up - coronal Cobb angle of main thoracic curvature immediately after operation.

Transverse diameter of pedicle: the place with the smallest transverse diameter on the coronal plane of pedicle.

Transverse diameter of pedicle costal head combination: the place with the smallest transverse diameter on the coronal plane of pedicle costal head.

### 2.6. Surgical Technique

All cases were treated with freehand nail placement technique, which was proposed by [19]. Cases with severe deformity were monitored by neuroelectrophysiology.

## 3. Experimental Results and Observation

### 3.1. Results of Pedicle Classification

Among various scoliosis deformities, the rate of pedicle deformity is shown in Table 1 and Figure 3, and type B stenosis deformity is more common. Type C atherosclerosis is the second, type E deformity is rare in idiopathic scoliosis, and type D and type E severe pedicle deformities are more common in neurofibromatosis scoliosis than idiopathic scoliosis.

### 3.2. Comparison of Deformity Rate: 21′

*X* ^2^ Test and Fisher's exact probability method were used for statistical analysis to analyze the difference between the thoracic and lumbar pedicle deformity rate of neurofibromatosis scoliosis and the thoracic and lumbar pedicle deformity rate of idiopathic scoliosis. The results are shown in Table 2. The difference in deformity rate between the two is statistically significant.

### 3.3. Screw Misplacement Rate

Of the 142 screws implanted in the neurofibroma group, 88 screws were found to be in good position through postoperative CT analysis and three-dimensional reconstruction, which met the grade 0 and grade 1 of Lee evaluation scheme: the screws were completely in the pedicle or the part penetrating the pedicle was less than 25% of the screw diameter. The other 54 screws were broken through the pedicle, which reached 25%∼50% of the screw diameter, or the broken pedicle was greater than 50% of the screw diameter. Therefore, the screw misplacement rate was 38.02%, and the screw placement satisfaction rate was 61.98%. Among the 111 screws placed in patients with idiopathic scoliosis, 86 screws were in a good position, 25 screws belonged to grade 2 or grade 3, the screw misplacement rate was 22.52%, and the screw placement satisfaction rate was 77.48%. Typical performance can be seen in Figure 4.

### 3.4. Transverse Diameter of Pedicle and Transverse Diameter of Pedicle Rib Combination

The transverse diameter of the pedicle in the AIS group was 2.73∼8.33 mm, which changed with segments. The transverse diameter of the T12 pedicle was the largest and the T4 pedicle was the smallest, which was only 1.77 mm. The transverse diameter of the scoliosis concave side in AIS patients was significantly smaller than that of the convex side. The transverse diameter of the thoracic pedicle rib complex in the AIS group is 10.04–14.91 mm. The measurement method is shown in Figure 4, and the transverse diameter gradually decreases from T1 to T5. The transverse diameter of the pedicle in the NF group was 1.57 mm∼8.21 mm, and the transverse diameter of the thoracic pedicle rib complex was 8.43–14.55 mm, which was less than that in the AIS group and shown in Figure 5.

Evaluation of the therapeutic effect of the patients with neurofibromatosis scoliosis on the coronal plane (see Table 3). The Cobb angle of the coronal plane of the main curve was 46°–126° (average 68.6°) before the operation, and the flat film was checked in time after operation for 4–58° (average 28.8°), the postoperative correction rate was 34%–92.5%, and the average correction rate was 58.8%. At the last follow-up, the Cobb angle of the main curve of the patients with neurofibromatosis group was 4°–62°, the correction rate was 34% − 92.5, and the average correction rate was 55.3%. Statistical analysis (see Table 4) shows that the effect of postoperative correction is accurate, the effect is accurate after the last follow-up (*P* < 0.01), and there is loss of correction (*P* < 0.01).

The evaluation of the therapeutic effect on the coronal plane of patients in the idiopathic scoliosis group is seen in Table 5. The Cobb angle of coronal plane of the main curvature before the operation was 28°–103° (average 61.4°), and the plain film was checked in time after the operation was 4–57° (average 22.4°), the postoperative correction rate was 35%–86.7%, and the average correction rate was 66.9%. At the last follow-up, the Cobb angle of the main curvature in the idiopathic scoliosis group was 4°–57°, and the correction rate was 31.3%–86.7%. The average correction rate was 64.2%.

There was no failure of internal fixation such as broken nails and rods in the two groups at the last follow-up. There were no neurovascular complications in the idiopathic scoliosis group. There was one case of postoperative total paralysis of both lower limbs in the neurofibroma group. The preoperative Cobb angle was 126°, only mild thumb motor function remained, and the level of sensory disturbance was in the perineum. There was no significant improvement in symptomatic treatment such as hormone shock after the operation. Serious neurological complications were considered. Internal fixation was taken out after X-ray reexamination, and the follow-up was unknown.

### 3.5. Typical Cases

A typical case is a 13-year-old male patient. Because of the “discovery of spinal deformity for 2 years,” I came to the outpatient department of our hospital. The outpatient department found that the thoracic 12 vertebral body was bent to the left, the X-ray showed scoliosis, and the Cobb angle was 60 degrees. The outpatient department originally planned to enter the ward with idiopathic scoliosis, and multiple milk coffee spots were found on admission. The diagnosis was as follows: (1) scoliosis deformity and (2) neurofibromatosis. The imaging data are shown in Figures 6 and 7.

## 4. Discussion and Analysis

Previous studies mainly focused on the diameter, angle, and treatment effect of the pedicle in normal young people or patients with idiopathic scoliosis. There are few reports on the overall shape of the thoracic pedicle in patients with neurofibromatosis. Lenke took the lead in observing the shape of the pedicle and divided it into four types: A, large cancellous bone lumen; B, small cancellous bone lumen; C, cortical bone lumen; D, no cortical lumen. Fu Changfeng and others made a further supplement after detailed measurement and analysis of the pedicle CT of 1440 thoracic vertebrae with various scoliosis types. Diameter <3 mm was selected as the criterion for pedicle stenosis. The consistency and reliability of typing are improved. At the same time, pedicle classification is closely combined with clinical practice. Type A pedicle can be inserted into pedicle probe without resistance, type B pedicle can be inserted into pedicle probe by hand close to the inner wall, type C pedicle needs to be hammered into pedicle because it cannot be inserted into pedicle probe by manual manipulation, and type D pedicle needs to be inserted into pedicle probe by pedicle bypass method. When an E-type pedicle appears, it should be considered to give up screw placement. The results showed that the morphological types of the pedicle of neurofibromatosis were a, B, C, D, and E, accounting for 44.61%, 37.53%, 8.92%, 7.08%, and 1.83%. The total deformity rate of the pedicle was 55.39%. There was a significant difference in the incidence of thoracic pedicle deformity between neurofibromatosis scoliosis and idiopathic scoliosis. Moreover, the pedicle was completely hardened, the incidence of absence was high, and screws could not be placed, indicating that neurofibromatosis scoliosis was more challenging, and better preoperative planning, intraoperative navigation, and monitoring measures were needed.

Thoracic pedicle screw fixation is potentially dangerous, especially in patients with neurofibroma and scoliosis. This paper also mentioned that, in this kind of patients, the vertebral body rotation in the top vertebral region is serious, the expansion of the dura mater and the expansion of the dura mater in the spinal canal are more likely to lead to dural sac tear, the morphological deformity of the pedicle is obvious, the degree of vertebral development is poor, and the distance between the spinal cord in the thoracic spinal canal and the medial edge of the pedicle is very limited, especially the concave side of the thoracic vertebra. Due to the inconsistent definition of poor screw placement, the misplacement rate of pedicle screws reported in the literature ranges from 2.5% to 72.4%. Although the reported manual screw placement techniques have different screw misplacement rates, and neurovascular complications are rare, the consequences are serious. In the neurofibromatosis patients in this study, there was a serious postoperative neurological impairment, manifested as total paralysis of both lower limbs and sensory impairment below perineum. In the AIS group, there was no neurovascular injury. Combined with the previous data, this is consistent with the efficacy and safety of posterior spinal fusion. The patients in the NF group are worse than those in the AIS group. In the face of NF patients, operators are more required to improve the accuracy of unarmed nail placement, use intraoperative nerve function monitoring equipment, improve the accuracy of nail placement with the help of intraoperative navigation and other auxiliary equipment, or make surgical templates by using three-dimensional reconstruction before the operation, so as to visually see the degree of spinal deformity of patients, so as to change the mode of operation or osteotomy.

The causes of screw misplacement may be various. The objective factors of pedicle deformity and vertebral rotation mentioned above will cause the misplacement of the pedicle screw. Subjectively, before screw placement, the operator needs to use the pedicle probe to deepen the screw path and probe to detect the integrity of the pedicle wall, while the postoperative CT and reconstruction show that the screw has penetrated the medial or lateral wall of the pedicle, which indicates that the probe and probe in the freehand screw placement technology are not completely reliable. In addition, some degree of operation in the orthopedic process, such as rotation, compression, and opening, may displace the implanted screws, form screw misplacement, damage blood vessels and nerves, or cause severe deformity in patients with NF, resulting in fracture during pedicle surgery, resulting in screw misplacement. Because this is a retrospective study, it is impossible to analyze whether the misplacement of pedicle screws is caused by objective pedicle deformity factors or surgical operation, which can be further studied.

## 5. Conclusion

In this paper, we have analyzed the arch root morphology, nail placement accuracy, degree of arch deformity, and three-dimensional Cobb angle in patients with NF scoliosis by CT 3D reconstruction. The results showed the following: (1) the rate of pedicle deformity in patients with neurofibromatosis scoliosis was high, and the deformity was more serious than that in patients with idiopathic scoliosis; (2) posterior vertebral fusion is effective in correcting neurofibromatosis scoliosis in coronal Cobb angle, but it is worse than idiopathic scoliosis; (3) patients with neurofibromatosis scoliosis have higher difficulty in screw placement, higher screw misplacement rate, and higher surgical risk. In addition, this study is a retrospective study with a small sample size, which needs to be further confirmed by large sample and multicenter randomized controlled trials.

In the future, we are interested to expend the proposed evaluation criteria to other groups of patients in different hospitals.

## Figures and Tables

**Figure 1:** Three-dimensional Cobb measurement.

**Figure 2:** Measurement of the internal diameter of vertebral arch and transverse diameter of vertebral arch and rib body.

**Figure 3:** Various types of pedicle morphology.

**Figure 4:** CT shows right side nail placement level 0 and level 3 left side nail placement level 2.

**Figure 5:** Transverse diameter of pedicle rib complex.

**Figure 6:** Milk coffee spot.

**Figure 7:** Preoperative examination.

**Table 1:** Types and deformity rates of the thoracolumbar pedicle in various scoliosis (%).

Side bend type	Type A	Type B	Type C	Type D	Type E	Deformity rate
	44.61	37.53	8.92	7.08	1.83	55.39
	89.85	31.97	7.02	1.16	0	40.15

**Table 2:** Comparison of pedicle deformity rate.

	*x* ^2^	*P* value
Comparison of two groups	4.51	0.024

**Table 3:** Evaluation of coronal efficacy in neurofibroma group.

Number	Preoperative coronal Cobb angle °	Postoperative Cobb angle °	Postoperative correction rate%	Cobb angle at the last follow-up	Follow-up correction rate%
1	71	16	77.4	23	67.6
2	50	33	34	33	34
3	51	25	50.9	27	47
4	93	47	49.1	47	49.4
5	82	52	36.5	60	27.5
6	55	19	65.5	19	65.5
7	53	4	92.5	4	92.5
8	92	36	60.8	41	55.4
9	54	29	40.6	41	55.4
10	45	22	51.1	25	44.4
11	126	58	56.3	58	56.3
12	73	42	42.4	44	39.7
13	58	9	84.5	13	77.4
14	85	33	61.2	35	58.9
15	46	8	82.6	10	78.3
15	68.6	28.8	58.8	31.3	55.3

**Table 4:** SPSS analysis of coronary curative effect in neurofibroma group.

Paired sample test						
Pairwise difference						
95% confidence interval of the difference						
	Mean value	Standard deviation	Standard error of the mean	Lower limit	Upper limit	*T*
For 1 preoperative Cobb angle, postoperative Cobb angle	39.75000	14.30851	3.57713	35.15554	47.37446	11.11215
For 2 preoperative Cobb angles, the last Cobb angle	37.31250	13.66123	3.41531	30.03295	44.59205	10.92515
For 3 postoperative cob angles, last Cobb angle	−2.43750	2.58118	0.64530	−3.81291	−1.06209	−3.77715
The postoperative correction rate of 4 cases, follow-up correction rate	3.53750	3.42926	0.85732	1.71018	5.36482	4.12615

**Table 5:** SPSS analysis of coronal efficacy in patients with idiopathic scoliosis.

Paired sample test						
Pairwise difference						
95% confidence interval of the difference						
	Mean value	Standard deviation	Standard error of the mean	Lower limit	Upper limit	*T*
For 1 preoperative Cobb angle, postoperative Cobb angle	39.06250	10.42733	2.60683	33.50617	44.61883	14.98515
For 2 preoperative Cobb angles, the last Cobb angle	37.37500	10.70125	2.67531	31.67271	43.07729	13.97015
For 3 postoperative cob angles, last Cobb angle	−1.68750	1.74045	0.43511	−2.61492	−0.76008	−3.87815
The postoperative correction rate of 4 cases, follow-up correction rate	0.776875	3.20369	0.80092	1.06062	4.47588	3.45715

## Data Availability

The datasets used during the current study are available from the corresponding author on reasonable request.
